# Investigating Temporal Kinematic Differences Caused by Unexpected Stimulation during Gait Termination through the Waveform-Level Variance Equality Test

**DOI:** 10.1155/2022/4043426

**Published:** 2022-07-04

**Authors:** Xi-ang Shen, Xuanzhen Cen, Yang Song

**Affiliations:** ^1^Department of Physical Education, Ningbo University of Finance and Economics, Ningbo 315175, China; ^2^Doctoral School on Safety and Security Sciences, Óbuda University, Budapest 1034, Hungary; ^3^Faculty of Engineering, University of Szeged, Szeged 6720, Hungary

## Abstract

The efficacy of the variance equality test in steady-state gait analysis is well documented; however, temporal information on where differences in variability occur during gait subtasks, especially during gait termination caused by unexpected stimulation, is poorly understood. Therefore, the purpose of the current study was to further verify the efficacy of the waveform-level variance equality test in gait subtasks by comparing temporal kinematical variability between planned gait termination (PGT) and unplanned gait termination (UGT) caused by unexpected stimulation. Thirty-two asymptomatic male subjects were recruited to participate in the study. A Vicon motion capture system was utilized to measure lower extremity kinematics during gait termination tasks with and without unexpected stimulation conditions. The *F*-statistic for each interval of the temporal kinematic waveform was compared to the critical value using a variance equality test to identify significant differences in the waveform. Comparative tests between two types of gait terminations found that subjects may exhibit greater kinematics variance in most lower limb joints during UGT caused by unexpected stimulation (especially at stimulus delay and reaction phases). Significant greater variances during PGT were exhibited only in the MPJ sagittal and frontal planes at the early stimulus delay phase (4-15% and 1-15%). This recorded dataset of temporal kinematic changes caused by unexpected stimuli during gait termination is essential for interpreting lower limb biomechanical function and injury prediction in relation to UGT. Given the complexity of the gait termination task, which involves both internal and external variability, the variance equality test can be used as a valuable method to compare temporal differences in the variability of biomechanical variables.

## 1. Introduction

Gait is the essential behavioral characteristic for quadrupeds represented by humans to move on solid substrates. Since this process involves a complex interplay of the nervous, musculoskeletal, and cardiovascular systems, any disorder of body function may affect gait performance [1]. By quantifying biomechanical characteristics during gait, pathological movement patterns can be evaluated. This crucial clinical method could also assess patient progress during rehabilitation and recovery from the influences of neurologic disease, musculoskeletal injury, or amputation of a lower limb [2–4].

Similar to physiological signals, most of the measured values in gait analysis (e.g., joint angles, joint moment, and ground reaction force) are not constants but fluctuate over time, varying from one stride to another [5]. Due to the existence of a fine-tuning system that regulates gait, the fluctuation between individual strides is relatively controlled, and the coefficient of variation reflected in gait parameters is also relatively limited [5, 6]. However, many studies supported that motor control may be compromised when the systems regulating gait are disturbed uncontrollably, resulting in multiscale dynamics alterations [5, 7, 8]. The essential manifestation is significant “noisy” variations in gait characteristics [9, 10]. For example, intrinsic motor or postural control during walking may be disrupted due to age- or disease-related decline of the central and peripheral nervous systems, with significantly greater gait variability [7, 11].

Gait variability measures have been considered better predictors of decreased mobility than absolute gait measures (e.g., gait speed) [7, 10–12]. Various methods have been proposed to estimate the gait variability of biomechanical parameters, commonly expressed in clinical studies using coefficients of variation [13, 14]. Furthermore, when the coefficient of variation is applied to kinematic or kinetic parameters, it presents an overall measure of variability for the waveform. However, this discrete measure provides little information about the timing of where differences in variability occur between groups. In a previous study, Kowalski et al. [13] proposed a waveform-level variance equality test based on a one-dimensional group waveform variance function to identify temporal differences in continuous variables and demonstrated its effectiveness by comparing ground reaction force variability during steady-state walking between young and old adults. This test for variance equality might provide a valid approach for comparing temporal differences in variances for other biomechanical variables, populations, and gait tasks.

Conventional gait tasks, such as walking and running, are continuous from initiation to termination, with the essential requirement to complete body movement while maintaining stability [15–17]. The balance would be challenged in gait subtasks that include initiation and termination, involving transitions from one statically stable or dynamically stable movement pattern to another [16]. In contrast to periodic steady-state gait, gait termination is a transient phenomenon that requires bilateral regulation of ground reaction forces for acceleration and deceleration using inter-limb coordination to stop the forward momentum and dissipate kinetic energy [18–20]. Designing gait termination models in clinical gait experiments has proven to be advantageous because the task can challenge both feedforwards, i.e., planned gait termination (PGT), and neuromuscular feedback control, i.e., unplanned gait termination (UGT) [21, 22]. The urgency of spontaneous activation of dynamic stability is exacerbated when people are forced to perform UGT in the face of unexpected stimulation [17]. Compared to PGT, the human body needs to increase braking force and decrease thrust for a short period to generate sufficient net braking impulse during UGT [23]. Many previous studies [17, 23, 24] have reported differences in biomechanical parameters between the two gait terminations. The results support that kinematic and kinetic fluctuations are significantly greater during gait termination induced by unknown stimuli (e.g., larger range of motion of lower extremity joint and larger regional plantar pressure) [17, 23, 24].

However, few studies estimate the variability of biomechanical variables during the two types mentioned above of gait termination. In particular, there is a lack of measurements that provide temporal information about where variability differences occur. Meanwhile, more information was required to verify further the efficacy of the waveform-level variance equality test in gait subtasks represented by gait termination. Given the research interest in temporal information on gait variability, the current study aimed to investigate temporal differences in group variance along the lower extremity kinematics waveform during PGT and UGT caused by unexpected stimulation through a waveform-level variance equality test. Combined with the importance of hip/knee extension and flexion strategies in stabilizing and performing stopping tasks during UGT [25], we hypothesized that subjects exhibited more significant kinematic variability in these two joints caused by unexpected stimulation during gait termination.

## 2. Materials and Methods

### 2.1. Subjects

Thirty-two participants were recruited to participate in this study, with ages of 23.63 ± 1.39 years, heights of 177.38 ± 5. 49 cm, weights of 67.97 ± 6.66 kg, and BMIs of 21.59 ± 1.70 kg/m^2^. The inclusion criteria were (i) adult male with dominant right leg; (ii) no musculoskeletal disorders that could potentially affect gait performance; (iii) no prior history of lower limb injuries or surgeries were reported in the first half of the year preceding data collection. Before the experiment, all subjects understood the study aim, requirements, and protocol and were thoroughly familiar with the procedures of experimental data collection. The Ethics Committee from the University (RAGH20201218) approved the study, and a written consent form was obtained from all individuals before participation.

### 2.2. Protocol

Each subject was instructed to perform gait termination trials randomly under two conditions: PGT and UGT, in the motion capture laboratory with normal indoor temperature and light. The gait trial protocol was consistent with the previously reported experimental procedure [23, 26]. Before data collection, they were asked to warm up and familiarize themselves with the collection environment for ten minutes. Moreover, at least three familiarization trials were completed for each gait termination task.

During the PGT trials, subjects were asked to walk barefoot along a 20 m walkway surrounded by eight infrared cameras. The gait activity was stopped when the participants reached a specific area within the walkway. Termination was established once the subject brought their feet together. For the UGT trials, subjects were not told beforehand which walkway area to stop in. Instead, they were given a termination signal during walking. The staff sent the termination instruction to the subjects by randomly ringing a bell. Participants needed to stop once they received the auditory signal delivered when their dominant foot stepped onto the walkway UGT area. To minimize the influences of anticipated sensory cues, twenty-five per cent of trials involved the termination signal, but the other seventy-five per cent did not. Each subject was required to provide six successful gait trial datasets, including three PGT and three UGT trials.

Kinematic data of the dominant lower extremity (right limb) joints was unilaterally measured via a three-dimensional motion capture system (Oxford Metrics Ltd., Oxford, UK) at a frequency of 200 Hz. Twenty-five reflective markers with a diameter of 9.0 mm were placed in each subject wearing tight-fitting pants to define the anatomical coordinate system and the center of the lower limb joint, including the hip, knee, ankle, and metatarsophalangeal joint. Based on a previous study [23], the pelvis, thigh, shank, forefoot, and rearfoot segments were built using double-sided tape to attach to the anatomical landmarks. The metatarsophalangeal joint angle was defined as an angle between the fore and rearfoot coordinate systems [27].

### 2.3. Data Processing

Experimental data of each gait termination trail during the stance phase were processed and analyzed in Visual 3D software (C-Motion Inc., Germantown, MD, USA) from C3D files created by Vicon Nexus Software (Vicon Motion System Ltd., Oxford, UK). A second-order low-pass Butterworth filter filtered the trajectory of reflective markers with a cut-off frequency of 10 Hz [28]. The joint angles were calculated by an inverse kinematics algorithm and normalized to 101 time points. Kinematic data of interest included the lower limb joint angles (hip, knee, ankle, and metatarsophalangeal joint) in the three motion planes (sagittal, frontal, and transverse phases) during the stance phase of two types of gait terminations. The stance phase of gait terminations was divided into the following three gait subphases: stimulus delay phase (0 ~ 38% of stance), reaction phase (39~65% of stance), and residual stance phase (66~100% of stance) [16, 26].

### 2.4. Statistical Analysis

Temporal differences in group variance along the lower extremity kinematics waveform during PGT and UGT caused by unexpected stimulation were investigated in this study. Due to the one-dimensional time-varying characteristic of the lower limb kinematics data, statistical analysis applied a waveform-level variance equality test proposed by Kowalski et al. [13]. Based on the open-source one-dimensional statistical parametric mapping (SPM 1d) package, the variance equality test employs the one-dimensional group waveform variance function to allow an *F*-test to compare group variances across an entire waveform [13, 29].

The *F*-statistic was calculated by dividing the group with the bigger variance by the group with the smaller variance, forcing the *F*-test into a right-tailed test [13]. *F*-critical was calculated as an inverse survival function of the *F* distribution with alpha (0.05), degrees of freedom, the number of discrete field nodes, and the field smoothness as inputs by the one-dimensional random field theory [13, 30]. All waveform-level variance equality tests were repeated at each time-point interval along the waveform using a custom script in MATLAB R2016a (The MathWorks, Natick, MA, USA).

## 3. Results

Figure 1 exhibits hip angle curves and waveform variances in sagittal, frontal, and transverse planes during two types of gait termination. In the sagittal plane, subjects had significantly greater hip flexion angle variability during whole UGT (0-100%) compared with PGT. The variance of hip adduction and abduction angles significantly increased in the sagittal plane at the stimulus delay phase and reaction phase during UGT (0–8% and 16-61%). In the transverse plane, significant differences in the kinematical variance between the two types of gait termination were exhibited only in the reaction phase (26-39%), and a greater external rotation value of the hip was found during gait termination caused by unexpected stimulation.

Knee angle curves and waveform variances in three motion planes during gait terminations are reported in Figure 2. In the sagittal plane, compared with PGT, extension variance was significantly greater at the stimulus delay phase, reaction phase, and early residual stance phase during UGT (3-9% and 16-81%). At a similar stage, variance in knee flexion angle in the sagittal plane was significantly greater during gait termination caused by unexpected stimulation (3-86%). Moreover, in the transverse plane, subjects also presented significantly greater knee internal rotation angles (5-9%, 15-75%, and 87-95%).

Figure 3 shows ankle angle curves and waveform variances in sagittal, frontal, and transverse planes during gait terminations. Compared with PGT, the stimulus delay phase (5-12%) and reaction phase (26-57%) present a greater variance in ankle plantar flexion angle during UGT in the sagittal plane. Kinematical variance in ankle inversion and external rotation were significantly greater during UGT in the frontal plane (4-9%, 15-36%, and 66-86%) and transverse plane (11-15%, 30-89%, and 96-100%), respectively.

MPJ angle curves and waveform variances in sagittal, frontal, and transverse planes during two types of gait terminations are reported in Figure 4. Compared with UGT, MPJ dorsiflexion and inversion angle variance were significantly greater at the stimulus delay phase of PGT in the sagittal plane (4-15%) and frontal plane (1-15%), respectively. However, subjects had significantly smaller MPJ external rotation variability during gait termination without unexpected stimulation (12-76%).

## 4. Discussion

Investigating the temporal kinematic differences between the two gait terminations might provide further insight into the biomechanical mechanisms of stopping gait induced by unplanned stimuli. The primary objective of this study was to explore temporal differences in group variance along the kinematics waveform of lower extremity joints during PGT and UGT caused by unexpected stimulation through the waveform-level variance equality test. In general, our hypotheses were partially correct, as some subjects exhibited greater kinematic variances in most lower limb joints (e.g., hip, knee, and ankle) during UGT caused by unexpected stimulation (especially at stimulus delay and reaction phases). In contrast, significantly greater variances during PGT have been exhibited only in the MPJ sagittal and frontal planes at the early stimulus delay phase.

Previous findings [23, 31] suggest that hip and knee kinematic information is the primary interest variable for gait termination tasks. Ridge et al. [31] reported that subjects exhibited greater knee and hip flexion throughout UGT than PGT. This hip/knee strategy can be explained by the subject needing to rely more on the knees and hips to absorb forces and control the movement of the center of mass to safely and quickly complete the gait termination task due to the unexpected stimulus. Nevertheless, considering that discrete analysis might compromise the spatiotemporal integrity of the original field, the approach of checking the entire stance phase than discrete parameters proved to be more suitable for determining biomechanical differences [32]. Therefore, the present study introduced a variance equality test that compares the temporal kinematics variance along the entire waveform of lower extremity joints to detect significant differences in variance [13]. Comparative analysis of the two types of gait termination tasks found that subjects showed greater variances in hip and knee joint kinematical data on three motion planes during UGT (especially at stimulus delay and reaction phases), which further supports previous research findings. The stimulus delay phase is a critical period, as subjects are judged by whether or not they receive an unexpected stimulus to perform the appropriate gait termination strategy. Once the subject receives the termination signal during this phase, the body will take a series of adjustments to generate a net braking impulse by increasing the initial braking impulse, attenuating postural instability, and avoiding falls. For example, the activity of the soleus amplitude was increased to slow tibial advancement, and the tibialis anterior and gluteus medius was increased to limit plantar flexion and maintain limb extension [33]. In addition, the significantly greater variability in hip and knee kinematics caused by unexpected stimuli during gait termination may also be due to the different termination strategies adopted by the subjects. A previous study [25] found that subjects' most typical stopping strategies were to flex the hips and stabilize in a position close to the peak hip flexion angle; the other strategy was to flex quickly and then return to a more extended position.

As a multisegmental system, the movements of the hip, knee, and ankle joints are linked with the lower extremity kinetic chain [23, 34]. In addition to the hip and knee differences discussed above, significantly greater ankle kinematic variance during UGT was presented in this study. Variability differences in the stimulus delay phase may be related to ankle plantar flexion and inversion during the process. Considering previously explored foot balance differences between two types of gait termination, this may result in gait imbalance and an increased risk of joint damage [17]. The MTJ, as an essential contributor to the energetics of the lower limb, needs to absorb energy and produce little or no energy during the pre-gait termination, i.e., stimulus delay and reaction phases [23, 35]. Notably, PGT shows significantly greater variability in the MPJ angle in the sagittal and frontal planes. In particular, the variance of MPJ dorsiflexion in the sagittal plane (4-15%) increased significantly during the stimulus delay phase of UGT. This may involve an integrated response regarding the MPJ-ankle coordination pattern to compensate for increased ankle dorsiflexion [23, 26].

Considering that gait termination may be challenging for the elderly and patients with balance disorders [16, 19–22, 36], particularly while facing unexpected stimulation, the location information on where differences in variability occur during gait termination may be critical [13]. For example, if excessive variability occurs in the frontal plane of the ankle during the stimulus delay phase, it may lead to an increased risk of ankle sprain [23, 37–39]. In addition, to improve the gait termination ability of patients with physiological or neurological diseases, the temporal kinematics of gait termination in asymptomatic subjects should be understood [31]. This dataset from the present experiment provides normative data describing the underlining mechanisms used to perform PGT and UGT caused by unexpected stimulation.

While acknowledging the results of this study, some limitations should be considered. Firstly, this study only compared the variability in the kinematics of lower limb joints and did not analyze the intrinsic kinematics or even the joint kinetics. Secondly, in the present study, all subjects were healthy young males, which resulted from the motivation to alleviate gender- and age-related differences in locomotion function. Lastly, the validity of the waveform-level variance equality test may not be fully verified by the results alone.

## 5. Conclusions

The sources of variability in gait measurement can be divided between the individual internal and environmental external [13]. Gait termination involves a complex neurological integration of different inputs, including sensory, vestibular, and proprioceptive [16]. Therefore, the analysis of gait variability during gait termination is complex, as both internal and external variability is involved. The present study conducted a prospective exploration into the temporal kinematic differences caused by unexpected stimulation during gait termination through a waveform-level variance equality test. The focus and attention of future research should be considered to further validate its validity by comparison with other gait variability methods, such as coefficient of variation and multiple correlation coefficients.

## Figures and Tables

**Figure 1:** Hip angle curves and waveform variances in sagittal, frontal, and transverse planes during planned gait termination (PGT) and unplanned gait termination (UGT). Note: shaded red vertical bars indicate the percentage range of stance phase where the variance during UGT was significantly greater with *p* < 0.05.

**Figure 2:** Knee angle curves and waveform variances in sagittal, frontal, and transverse planes during planned gait termination (PGT) and unplanned gait termination (UGT). Note: shaded red vertical bars indicate the percentage range of stance phase where the variance during UGT was significantly greater with *p* < 0.05.

**Figure 3:** Ankle angle curves and waveform variances in sagittal, frontal, and transverse planes during planned gait termination (PGT) and unplanned gait termination (UGT). Note: shaded red vertical bars indicate the percentage range of stance phase where the variance during UGT was significantly greater with *p* < 0.05.

**Figure 4:** Metatarsophalangeal joint (MPJ) angle curves and waveform variances in sagittal, frontal, and transverse planes during planned gait termination (PGT) and unplanned gait termination (UGT). Note: shaded red and black vertical bars indicate the percentage range of stance phase where the variance during UGT or PGT was significantly greater with *p* < 0.05, respectively.

## Data Availability

The data presented in this study are available on request from the corresponding author. The data are not publicly available due to ethical considerations.
